# Ultrasound Images under an Optimized Image Processing Algorithm in Guiding the Neurological Safety of Resection of Lumbar Disc Nucleus Pulposus in Spinal Surgery

**DOI:** 10.1155/2022/3232670

**Published:** 2022-06-02

**Authors:** Kaiwei Yin, Yehai Chen, Shuying Gao

**Affiliations:** Department of Orthopedics, Dongyang Garden Tian's Hospital, Dongyang, Jinhua, 322100 Zhejiang, China

## Abstract

This study was aimed at investigating the effect of an optimized image processing algorithm in ultrasound images and the influence of resection of lumbar disc nucleus pulposus in spinal surgery under the guidance of ultrasound images on the neurological safety of patients. A total of 60 patients with lumbar disc herniation were selected and divided randomly into the control group and observation group. Patients from the control group were treated with resection of lumbar disc nucleus pulposus by an X-ray-guided foraminal microscope, and patients from the observation group underwent the ultrasound image-guided surgeries with an optimized image processing algorithm. Then, the treatment of patients from the two groups was compared. The results showed that the radiotherapy time in the control group was 120 ± 6.3 min and the radiotherapy dose was 129 ± 10.3 min/sec, while the radiotherapy time in the observation group was 4.5 ± 1.2 min and the radiotherapy dose was 22 ± 7.7 min/sec. The time and dose of radiotherapy in the observation group were significantly lower than those in the control group (*P* < 0.05). In the control group, the numbers of significant effective cases, effective cases, and ineffective cases were 8, 16, and 6, respectively, while those in the observation group were 12, 18, and 0, respectively. The comparison between the groups showed that the number of effective cases and the number of effective cases in the observation group were significantly higher than those in the control group, and the number of ineffective cases was significantly lower than that in the control group (*P* < 0.05). In conclusion, ultrasound-guided percutaneous foraminal lumbar discectomy could improve patients' clinical symptoms, promote clinical efficacy, and reduce postoperative pain symptoms, thereby accelerating the postoperative rehabilitation of patients. Moreover, it was extremely safe for the nerves.

## 1. Introduction

Lumbar disc herniation is a common disease in spinal surgery. With the rapid development of the economy and society, the pressure of adult life and work is increasing, the intervertebral disc gradually undergoes degenerative changes, and the fibers in the fibrous annulus become thicker and brittle and eventually break, so that the intervertebral disc loses its original elasticity and cannot bear the original pressure [1]. Under overwork, sudden changes in body position, vigorous action, or violent impact, the annulus fibrosus can bulge outwards, so that the nucleus pulposus can also protrude through the fissures of the ruptured annulus fibrosus, eventually forming a herniated disc [2]. Lumbar disc herniation can lead to waist pain, sciatic nerve radiating pain, numbness and pain in the lower limbs, hypoesthesia or allergies, muscle atrophy, thinning of the affected leg, and difficulty in walking. In severe cases, it can result in dysfunction of the urine and bowels, paralysis of the lower limbs, and long-term bed rest, thereby reducing the patient's quality of life and losing the ability to work. According to pathological changes and computed tomography (CT), magnetic resonance imaging (MRI), and other manifestations, lumbar disc herniation can be divided into four types, including bulging, protruding, free prolapse, and Schmorl's nodules [3].

The clinical treatment of lumbar disc herniation is generally divided into conservative treatment and surgical treatment [4]. Most patients can be relieved or cured by nonsurgical treatment. What is more, the principle of conservative treatment is not to restore the degenerated and herniated intervertebral disc tissue to the original position, but to change the relative position or partial return of the intervertebral disc tissue and the compressed nerve root to reduce the pressure on the nerve root, loosen the nerve root adhesion, and eliminate inflammation of nerve roots, thereby alleviating symptoms [5]. Nonsurgical treatment is mainly suitable for patients who are young with the first attack or a short course of the disease, suffer from mild symptoms that can be relieved after rest [6], and had no obvious spinal stenosis on imaging examination. However, surgical treatment is for patients who have a medical history of more than three months, have ineffective or effective strict conservative treatment, often relapse and suffer from severe pain with the first onset, had a severe pain, especially in the lower limb obvious symptoms, are difficult to move and sleep, are in a forced position, and are complicated with spinal stenosis. Moreover, surgical treatment can also be divided into open surgery and minimally invasive surgery. Open surgery refers to the removal of the nucleus pulposus through the posterior lamina fenestration, which mainly includes conventional nucleus pulposus and endoscopic nucleus pulposus. The technical effect of open surgery is clearer, but there are also more significant drawbacks. It can cause mechanical damage to the spine, destroy the stability of the spine, and damage the soft tissues around the spine. It leads to increased bleeding and higher requirements for the surgeon. The nerve needs to be stretched during the surgery and may cause nerve damage, and it is easy to form spinal dural scar adhesion during the postoperative recovery process, which seriously hinders the postoperative recovery process [7].

In recent years, with the development of science and technology, imaging technology in the field of biomedicine has also been advancing by leaps and bounds. Besides, with the development of spinal instruments and techniques, minimally invasive spinal surgery has become the main way of surgical treatment [8, 9]. The advent of modern endoscopic technology, three-dimensional imaging technology, and navigation technology has effectively promoted the development of minimally invasive spinal surgery. In order to obtain effective and clear lumbar anatomical images, ultrasound imaging technology and low-frequency ultrasound probes are required. Ultrasound imaging technology can also be applied to the anesthesia of the lumbar spine, which is especially beneficial for patients with a relatively obese body [10]. In addition, the image optimization processing algorithm was also adopted in this study. After ultrasound imaging, the optimization model was established to realize the global optimization restoration of the images. What is more, the image segmentation was performed to display the key parts by magnification, thereby realizing the optimal image distribution [11]. In this study, patients with lumbar disc herniation were selected for ultrasound image monitoring, and an optimized image processing algorithm was employed to analyze and sort out, aiming at exploring the neurological safety of resection of lumbar disc nucleus pulposus.

## 2. Materials and Methods

### 2.1. Research Objects

Sixty patients with lumbar intervertebral disc herniation were selected as the research objects, who were admitted to the hospital from March 2018 to January 2020. Besides, they received surgical treatment. According to the random number table, they were rolled into the control group and the observation group, with 30 cases in each. Patients from the control group were guided by X-ray, with 19 males and 11 females. They were 38-75 years old, with an average age of 56.59 ± 3.17 years. The body mass index (BMI) was 17-24 kg/m^2^, with an average of 20.01 ± 1.15 kg/m^2^. In the observation group, the image optimization processing algorithm was adopted under the guidance of ultrasound imaging. There were 20 males and 10 females, and they were 36-74 years old, with an average age of 55.03 ± 3.22 years. The BMI was 17.21-23.81 kg/m^2^, with an average of 20.31 ± 1.02 kg/m^2^. There was no statistically great difference in the general data of patients from the two groups, such as gender, age, and BMI (*P* > 0.05), and the groups were comparable. This study had been approved by the ethics committee of the hospital, and informed consent was obtained from patients.

Inclusion criteria are as follows: patients with recurrent low back and leg pain, and the degree of leg pain was more severe than the degree of low back pain; those with paresthesia in some areas of the lower extremities; patients with at least one of below three signs: the straight leg raising test was less than 50°, the strengthening test was positive, and the healthy side raising test was positive; and patients with at least two of below signs: muscle atrophy, muscle weakness, paresthesia, and reflex changes.

Exclusion criteria are as follows: those with mental illness and unable to communicate and communicate effectively with the researchers; those who are allergic to the drugs used in this work; patients with systemic or local infection; patients with severe spinal degeneration and instability; patients with obvious posterior longitudinal ligament calcification and fibrocartilaginous plate ossification; patients with severe structural abnormalities of the lamina, facet joints, and spinal canal; and patients with dysfunction of important organs, severe systemic diseases, and inability to tolerate surgery.

### 2.2. Methods

#### 2.2.1. Image Optimization Processing Algorithm

The image optimization processing algorithm included image reconstruction, image enhancement, and edge detection. In the image reconstruction process, the filter operator could be optimized to reduce the impact of projection noise on the reconstruction result, and high-resolution images could be reconstructed to eliminate and reduce the effect of mixing. When performing image reconstruction, a certain pixel value of the low-resolution image needed to be weighted, which could be expressed as follows.

(1) $$\begin{array}{c} A_{m,n}=\overset{P}{\underset{s=1}{\sum }}Q_{m,n,s}X_{s}+l_{m,n}. \end{array}$$

In Equation (1), *m* = 1, 2, 3⋯, *n* = 1, 2, 3⋯; and *P* = *l*2*m*; *A*_*m*,*n*_ represented the element in the *n*-th frame, the weighted value *Q*_*m*,*n*,*s*_ stood for the *s*-th high-resolution pixel for the contribution of the pixel value of the *n*-th frame, and *l*_*m*,*n*_ expressed the influence of the additional noise on the pixel value of the *n*-th frame. In order to estimate low-resolution images, a regularized cost function *Y*_(*x*)_ needed to be carried out, and the solution that minimized the cost function was required, as shown in the following equation.

(2) $$\begin{array}{c} Y_{\left(x\right)}=\frac{1}{2}\overset{mn}{\underset{m=1}{\sum }}{\left(f_{m}-\overset{P}{\underset{S=1}{\sum }}Q_{m},x_{1}\right)}^{2}+\frac{q}{2}\overset{P}{\underset{d=1}{\sum }}{\left(\overset{P}{\underset{j=1}{\sum }}l_{j},x_{j}\right)}^{2}. \end{array}$$

In image enhancement, some information in an image could be highlighted according to specific needs, while some unwanted information could be attenuated or removed. In the operation process, the equations that needed to be adopted were as follows.

(3) $$\begin{array}{c} W\left({\text{g}}_{\text{i}}\right)={\left\|b-{jg}_{i}\right\|}^{2}, \end{array}$$

(4) $$\begin{array}{c} D_{\left(gi\right)}=\frac{\sum_{gi-m}^{n}\sum_{gi-n}^{m}X_{\left(i+m\right)\left(i+n\right)}}{m\times n}. \end{array}$$

In Equations (3) and (4), *D*_(*gi*)_ stood for mutation operation, *g*_*i*_ meant the inferred restored image represented by the individual *i*, *b* represented the observed degraded image, and *j* expressed the point spread function in the degradation process.

Image segmentation was to use the gray features of the image to select the best threshold, to divide the pixels in the image, and to perform coding and edge detection. The marginal monitoring error *f*_(*x*, *y*, *e*)_ could be calculated as the following.

(5) $$\begin{array}{c} f_{\left(x,y,e\right)}=\overset{x}{\underset{e=1}{\sum }}{\left(\sqrt{{\left(x_{e}-x\right)}^{2}+{\left(y_{e}-y\right)}^{2}}-e\right)}^{2}. \end{array}$$

In Equation (5), (*x*, *y*) stood for the edge coordinates. Among the edge points obtained by image processing, they would be disturbed by noise points, in which wpi;d affects the measurement accuracy. Therefore, the above equations were required.

#### 2.2.2. Imaging Guidance Method

X-ray-guided percutaneous vertebral disc nucleus resection through a foraminal approach was as follows. First, there were disc puncture and discography, and the patient was in the prone position. The front and side positions of the C-arm machine were positioned on the affected joint, and then the red pen was used to mark. The puncture point was determined according to the lesion space and the patient's physical condition. A local anesthetic was injected into the patient, and the contrast agent was administered at the same time. The lesions of the intervertebral disc were observed through fluoroscopy. Next, a working channel was needed to be placed in the formed intervertebral foramen, and a guide rod and a dilator were placed in sequence to prepare the working channel through the application of a surgical system. The nucleus pulposus removal and decompression were performed under the field of the endoscope, and the endoscopic special nucleus pulposus clamps, probes, and other instruments were used for surgery. When nerve roots were exposed, flexible bipolar radiofrequency electrocoagulation was used to ablate the nerve endings that grew into the annulus fibrosus. The nerve endings in the ring were ablated. At the end of the surgery, the position of nerve tissue and ligament tissue needed to be confirmed under the microscope, and the surgery could be ended when there was no obvious bleeding in the surgical field. After the surgery, anti-infection and anti-inflammatory treatments were required, the waist circumference was fixed on the first day after the surgery, and the patient was asked to perform under-bed activities to prevent nerve root adhesion.

There was the ultrasound image-guided percutaneous transforaminal lumbar disc nucleus resection based on the optimized image processing algorithm. An ultrasonic cross-sectional examination of the lumbar spine was performed to determine the position of the spinous process, the midline of the lumbar spine, and the segment of the lumbar spine. During the examination, the long axis of the ultrasound ray was along the direction of the spinous process line, the longitudinal axis was placed on the posterior midline, and below the ultrasound hyperechoic line was the spinous process, where the position of L5 was accurately located. Then, the probe was moved outwards to determine the lumbar space and other anatomical positions. In the imaging process, the image optimization algorithm was used to process, and then, the C-arm machine was positioned anteriorly and laterally at the diseased joint, which was marked with a red pen. Besides, the puncture point was determined according to the gap of the disease and the patient's physical condition. Next, the patient was injected with an anesthetic, and the probe was used for puncture. When exploring along the long axis of the puncture needle in the direction of the facet joint, a linear hyperechoic signal could be seen under a mass-like hypoechoic area, or a thin anechoic linear structure interruption indicated that the puncture needle reached the facet joint. Then, the ultrasound probe was employed to take a longitudinal section parallel to the midline of the posterior midline, and the joint position of the puncture needle can be clearly observed. Moreover, the nucleus pulposus was performed with endoscopy, and the anti-infection and anti-inflammatory treatment was also required after surgery.

### 2.3. Observation Indicators

First, the baseline data of patients from the two groups were compared.

Second, the average radiation time and the radiation dose to the neck of patients from the two groups were compared.

Third, the internal dose, surface dose, and effect dose of the lead coating were compared under the guidance of the two images.

Fourth, the imaging examination images of patients from the two groups were compared.

Fifth, the surgical time of patients from the two groups was compared.

Sixth, the clinical efficacy of patients from the two groups was compared, referring to the relevant criteria. Besides, the marked effect meant that the postoperative straight leg elevation could increase by more than 30% before treatment, but it was still less than 70%. The effective effect indicated that the straight leg elevation was less than 30%. In addition, there was no effect if the patient had no improvement or even worsened after treatment.

Seventh, the postoperative pain scores of patients from the two groups were compared, the visual analogue scale (VAS) was used for evaluation, and the range was 0-10 points. The higher the score, the more severe the pain. The detailed scoring criteria are shown in Figure 1.

### 2.4. Statistical Methods

The SPSS 21.0 statistical software was used for data analysis, measurement data were expressed by *x̅*±*s*, and *t* test was performed. Besides, the count data were expressed by case (%) and detected by *x*^2^. In addition, *P* < 0.05 indicated that the difference was statistically substantial.

## 3. Results

### 3.1. Comparison on the Baseline Data of Patients from the Two Groups

The comparison results of the general data of the two groups of patients are shown in Figures 2–4. They illustrate that the control group included 19 male patients and 11 female patients, the average age of the patients was 56.59 ± 3.17 years old, and the average BMI of the patients was 20.01 ± 1.15 kg/m^2^. The observation group included 20 male patients and 10 female patients, with an average age of 55.03 ± 3.22 years old and an average BMI of 20.31 ± 1.02 kg/m^2^. There was no significant difference in general data such as gender, age, and BMI between the two groups (*P* > 0.05).

### 3.2. Comparison on the Average Radiation Time and the Radiation Dose of the Neck of Patients from the Two Groups

The comparison results of the average radiotherapy time and radiotherapy dose for the neck of the two groups of patients are shown in Figure 5. The radiotherapy time in the control group was 120 ± 6.3 min, and the radiotherapy dose was 129 ± 10.3 min/sec, while those in the observation group were 4.5 ± 1.2 min and 22 ± 7.7 min/sec, respectively. The time and dose of radiotherapy in the observation group were significantly lower than those in the control group (*P* < 0.05).

### 3.3. Comparison on the Lead Coating Surface Dose, Internal Dose, and Effect Dose under the Guidance of Two Imaging Methods

The comparison results of the surface dose, internal dose, and effect dose of lead coating in the two groups of patients are shown in Figure 6. It revealed that the surface dose, internal dose, and effect dose of lead coating in the control group were 15 ± 3.1 min/sec, 130 ± 9.3 min/sec, and 9 ± 1.4 min/sec, respectively, while those in the observation group were 2 ± 0.8 min/sec, 18 ± 2.6 min/sec, and 1.5 ± 0.3 min/sec, respectively. The comparison between groups showed that the surface dose, internal dose, and effect dose of lead coating in the observation group were significantly lower than those in the control group (*P* < 0.05).

### 3.4. Imaging Examination Images of Patients from the Two Groups

Through imaging examination, it revealed that the imaging under ultrasound guidance was clearer than the imaging under X-ray guidance, and the probe position was accurate, as shown in Figures 7–9.

### 3.5. Comparison on the Surgical Time of Patients from the Two Groups

The comparison results of the operation time of the two groups of patients are shown in Figure 10. The average operation time of the control group was 100 ± 10.3 min, and the average operation time of the observation group was 68 ± 5.7 min. The comparison between groups showed that the average operation time of the observation group was significantly shorter than that of the control group (*P* < 0.05).

### 3.6. Comparison on the Clinical Efficacy of Patients from the Two Groups

The comparison results of clinical efficacy of the two groups of patients are shown in Figure 11. In the control group, the number of significant effective cases, the number of effective cases, and the number of ineffective cases were 8, 16, and 6, respectively, while those in the observation group were 12, 18, and 0, respectively. The comparison between the groups showed that the number of effective cases and the number of effective cases in the observation group were significantly higher than those in the control group and the number of ineffective cases was significantly lower than that in the control group (*P* < 0.05).

### 3.7. Comparison on the Postoperative Pain Scores of Patients from the Two Groups

The comparison results of postoperative pain scores of the two groups of patients are shown in Figure 12. The postoperative pain score was 7.5 ± 1.6 points in the control group and was 3 ± 0.9 points in the observation group. Compared with the control group, the postoperative pain score of the observation group was significantly lower than that of the control group, and the difference was statistically significant (*P* < 0.05).

## 4. Discussion

With the development of biological technology, the surgical treatment of lumbar disc herniation has become more and more advanced [12]. The application of imaging technology in surgical treatment is a new type of treatment, and the X-ray-guided percutaneous foraminal endoscopic resection of lumbar disc nucleus pulposus by the foraminal approach has substantial advantages over traditional treatment methods [13]. It can use images to make the position of the probe more accurate, and the surgical access is safer, making the treatment of nucleus pulposus great progress. However, it has a greater negative impact on the surgeon and related personnel due to the high X-ray radiation dose, so there are clinical limitations [14, 15].

The percutaneous foraminal endoscopic resection of lumbar disc nucleus pulposus by the foraminal approach under the ultrasound guidance can obviously reduce the drawbacks of X-rays. This technology can obtain clearer images of the bony structure behind the lumbar spine and clearly show the anatomical positions of facet joints and paravertebral muscles [16]. Moreover, ultrasound technology can also display the specific location of soft tissues and puncture needles, thereby greatly avoiding the risk of puncture needles penetrating the parietal peritoneum and nerve tissues [17]. However, the image optimization processing algorithm was also employed in this study to make the ultrasound image clearer due to the deepness of the spine structure. The blurred, edge, and misaligned images were sorted and analyzed, and the location of the lesion and the surgical field could be displayed more clearly. The surgical field is more conducive to the development of surgery. The results of this study suggested that the average radiation time under ultrasound guidance, the radiation dose of the neck, and the surface dose of the leading coat, the internal dose, and the effect dose were all lower than those under X-ray guidance. Ultrasound-guided imaging was clearer than X-ray-guided imaging, and the precise location of the probe confirmed the advantages of ultrasound-guided imaging, which was similar to the results of most studies [18]. In addition, the surgical time of the observation group decreased steeply compared with the control group (*P* < 0.05). This is consistent with previous research results.

Ultrasound technology can play a greater role in the diagnosis and treatment of spinal diseases. There are also some scholars who apply the combination of CT and ultrasound-guided technology and percutaneous endoscopic lumbar discectomy by transforaminal approach, showing the advantages of ultrasound technology to guide this surgery [19]. The results of this study indicated that the number of markedly effective cases and effective cases of the observation group increased dramatically in contrast to the number of the control group (*P* < 0.05), while the number of ineffective cases was lower than that of the control group (*P* < 0.05). The postoperative pain scores of the observation group dropped steeply compared with the control group (*P* < 0.05). The results of Zhao et al. [20] showed that an ultrasound-guided percutaneous transforaminal approach for transforaminal lumbar discectomy can better the clinical symptoms of patients, improve clinical efficacy, and reduce postoperative pain symptoms; it was extremely safe for nerves and promotes postoperative recovery. This is consistent with the findings of this work.

## 5. Conclusion

The nucleus pulposus of the lumbar intervertebral disc in spinal surgery guided by the optimized image processing algorithm could clearly show the bony structure behind the lumbar spine, as well as the anatomical positions of the facet joints and paravertebral muscles. Besides, ultrasound technology could also display the specific location of soft tissue and puncture needles, improving the safety of nerve tissue. In addition, the image under ultrasound guidance was clearer than that under X-ray guidance, and the position of the probe was accurate, confirming the advantages of ultrasound guidance. The results of this study revealed that ultrasound-guided percutaneous foraminal lumbar discectomy could improve the patient's clinical symptoms, promote clinical efficacy, and reduce postoperative pain symptoms, which was extremely safe for nerves and could shorten the time for the patient to recover after surgery. It was believed that with the maturity of the combination of imaging technology and surgery and the rapid development of the image optimization algorithm, the application space of this technology in biomedicine had to be broader. The disadvantage of this study is that the sample size of the study is small, which will cause errors in the data of the research results. Therefore, it is necessary to expand the sample size for further research to obtain more scientific and reliable research data, providing an effective reference for clinical treatment.

## Figures and Tables

**Figure 1:** The detailed criteria for VAS.

**Figure 2:** Gender ratio of patients from the control group.

**Figure 3:** Gender ratio of patients from the observation group.

**Figure 4:** Comparison on the age and BMI of patients from the two groups.

**Figure 5:** Comparison on the average radiation time of the image and the radiation dose of the neck in patients from the two groups. (a) Average radiation time. (b) Radiation dose to the neck. ^∗^ means *P* < 0.05.

**Figure 6:** Lead coating surface dose, internal dose, and effect dose under the guidance of two imaging methods. (a) Lead coating surface dose. (b) Internal dose. (c) Effect dose. ^∗^ indicates *P* < 0.05.

**Figure 7:** Ultrasound-guided image.

**Figure 8:** Probe position under ultrasound guidance.

**Figure 9:** Image under X-ray guidance.

**Figure 10:** Comparison on the surgical time of patients from the two groups. (a) The control group. (b) The observation group. ^∗^ means *P* < 0.05.

**Figure 11:** Comparison on the clinical efficacy of patients from the two groups. (a) Marked effect. (b) Effective effect. (c) No effect.

**Figure 12:** Postoperative pain scores of patients from the two groups. (a) Control group. (b) Observation group. ^∗^ presents *P* < 0.05.

## Data Availability

The data used to support the findings of this study are available from the corresponding author upon request.
